The article "Long-Term Effect of Left Atrial Appendage Occlusion in Treating Patients with Previous Ischemic Stroke on the Disease Recurrence" was published in 2021. Journal: Comput Math Methods Med.

# Long-Term Effect of Left Atrial Appendage Occlusion in Treating Patients with Previous Ischemic Stroke on the Disease Recurrence

**DOI:** 10.1155/2021/6991002

**Published:** 2021-10-13

**Authors:** Jia Yu, Yufeng Liu, Peng Sun, Xing Guo, Haiyang Jiang, Wei Fang, Xin Jin

**Affiliations:** ^1^Department of Neurosurgery, Tangdu Hospital, Air Force Military Medical University, Xi'an, Shaanxi Province 710038, China; ^2^Department of Nursing, Tangdu Hospital, Air Force Military Medical University, Xi'an, Shaanxi Province 710038, China

## Abstract

**Methods:**

A total of 120 patients with IS admitted to Tangdu Hospital from July 2016 to September 2017 were grouped into the control group (*n* = 60) and the observation group (*n* = 60). Patients in the control group were only treated with thrombolytics and anticoagulants while those in the observation group were treated with both drugs and LAAO. Transesophageal echocardiography (TEE) was performed to observe the occlusion of LAA in patients in the observation group after 45 d and 6 months, respectively. Clinical outcomes in two groups were compared from the following aspects: recurrence of IS, incidence of systemic embolism, and the 3-year recurrence-free survival (RFS). The 3-year IS recurrence of patients was compared by Fisher's exact test.

**Results:**

No significant differences were observed at baseline levels (age, sex, etc.) between the observation group and control group (*p* > 0.05). During follow-up visit of 45 d and 6 months, all occluders met the efficacious occludsion criteria. The results of TEE at 45 d after LAAO showed that 50% of patients (30/60) in the observation group had complete occlusion of LAA. The results of TEE at 6 months after LAAO suggested that 58.3% of patients (35/60) had complete occlusion of LAA. IS recurrence in the observation group (3.33%, 2/60) was significantly lower than that in the control group (18.33%, 11/60), with the difference presenting statistical significance (*p* = 0.008). Incidence of systemic embolism in the observation group (1.67%, 1/60) was markedly lower than that in the control group (13.33%, 11/60) (*p* = 0.014). The average RFS in the observation group (31.97 months, 95% CI: 27.50~32.31 months) was notably longer than that in the control group (29.91 months, 95% CI: 29.85~32.92 months) (*p* < 0.05). The 3-year IS recurrence of patients between two groups compared by Fisher's exact test showed significant differences (1 year: *p* = 0.014, 2 year: *p* = 0.008, 3 year: *p* = 0.008).

**Conclusion:**

Regarding patients with previous IS who had poor response to thrombolytics and anticoagulants, LAAO could effectively decrease recurrence of IS and incidence of systemic embolism and prolong RFS of patients. LAAO was, therefore, an alternative for patients with high IS recurrence risk.

## 1. Introduction

Stroke, as the most prevalent angiocardiopathy, is one of the main causes of deaths and disabilities [1]. Ischemic stroke (IS), characterized by high recurrence [2], accounts for 75-80% of all stroke cases as the predominant subtype [3]. A study about IS recurrence unveiled that the 1-year cumulative recurrence rate of IS is 5.4% among prior IS patients, and the 5-year cumulative recurrence rate is 11.3% [4]. Compared with initial-onset IS patients, patients with recurrence have higher mortality and disability rates [5, 6]. Over 90% of stroke patients suffer from sequelae, with one-third of them unable to resume daily life activities as before [7], thereby imposing huge financial and mental burdens on their family. A cost-effectiveness study of IS intervention displayed that IS routine care costs for 13,940 RMB a year [8]. So far, some progresses have been made to assist patients in recovering from IS, with improvement in recanalization therapy using pharmacological and mechanical thrombolysis [9]. At present, drug interventions such as oral thrombolytics and anticoagulants are applied to patients with previous stroke, but some of them respond poorly to these drugs. Hence, intervention by left atrial appendage occlusion (LAAO) is warranted to reduce recurrence rate of IS.

LAA is a small pouch on left atrium (top left chamber of the heart), which forms during the fourth week of embryonic development [10]. In transesophageal echocardiographic (TEE) studies, over 90% of thrombi is found in LAA of patients with nonvalvular atrial fibrillation [11, 12]. LAAO is an interventional therapy. The guide wire is usually placed in LAA through puncture of femoral vein under local anesthesia, and then, the occluder is inserted. The occluder is capable of preventing thromboembolism and reducing risk of stroke, and thus, LAAO is considered an effective preventive therapy for thrombosis [13]. Multiple pieces of clinical research have verified the efficacy of LAAO in preventing nonvalvular atrial fibrillation stroke. Osmancik et al. [14] reported that regarding patients with high stroke risk and increasing bleeding risk, LAAO is noninferior to direct oral anticoagulants in prevention of major atrial fibrillation-related cardiovascular, neurological, and bleeding events. A network meta-analysis by Hanif et al. [15] revealed that LAAO appears to be the most efficacious avenue to stroke outcomes when compared to warfarin, aspirin, or placebo. A relevant study also pointed out similar safety outcomes between patients with stroke undergoing LAAO and those without LAAO, with notable decreases in stroke/transient cerebral ischemia, as well as major bleeding events during follow-up, suggestive of safety and efficacy of LAAO in patients with previous stroke [16]. Nonetheless, few investigations are about the impact of LAAO in treating patients with previous IS on disease recurrence.

This retrospective study analyzed efficacy and long-term effect of LAAO in treating patients with previous IS on disease recurrence, thus laying foundation for disease management.

## 2. Materials and Methods

### 2.1. Research Objects

A total of 120 patients with IS admitted to Tangdu Hospital from July 2016 to September 2017 were selected as research objects. LAA thrombi in the included patients were confirmed by echocardiogram. The patients included in the study had poor efficacy after receiving preventive treatments such as anticoagulants and thrombolytics. Patients were divided into the control group and the observation group according to therapeutic avenues. Patients in the control group (*n* = 60) were only applied with drugs such as thrombolytics, lipolytic drugs, and antiplatelet drugs according to their specific symptoms. Patients in the observation group (*n* = 60) underwent LAAO based on medication. This study was approved by the Medical Ethics Committee of Tangdu Hospital. All participants in the study provided the informed consent.

### 2.2. LAAO

LAAO was done on patients in the observation group under general anesthesia or local anesthesia. During the procedure, the LAA diameter and anchorage area were measured by TEE or intracardiac ultrasound. An appropriate Watchman occlude device was selected based on the shape of LAA and number of lobes. As in standard procedures, under real-time ultrasound guidance, the patient was subjected to femoral vein puncture, during which sheathing canal and puncture needle were inserted through vein in patient's upper leg, followed by conventional transseptal puncture. In detail, a sheath threaded through the interatrial septum via a needle puncture. Then, a guide wire was advanced to left superior pulmonary vein. Along the guide wire, the Watchman occluder sheath and a pigtail catheter were inserted into the vein. Through dual measurements by angiography and electrocardiogram, the applied size of occluder was determined. The occluder was inserted into the LAA via the sheath, and it was released to seal off the LAA. After the occluder was confirmed well-positioned without displacement during traction and the release coefficient was stable, the sheath was pulled out. The patient was transferred to the Cardiac Care Unit after LAAO.

### 2.3. Outcome Measures

Forty-five d and six months after the procedure, TEE study was used to determine whether the efficiency of LAAO met the position, anchor, size, and seal (PASS) criteria [17], with residual shunt ≤ 5 mm. Other outcome measures included the recurrence of IS, incidence of systemic embolism, and three-year recurrence-free survival (RFS) in the two groups after LAAO.

### 2.4. Follow-Up Visit

Forty-five d and six months after LAAO, patients in the observation group were reexamined by TEE to measure whether there was residual shunt in the LAA and thrombosis on surface of the occluder. During the 3-year follow-up visit, recovery of lesions, signs of thrombosis, and other adverse events in each group were examined by imageological paths every six months.

### 2.5. Statistical Analysis

Statistical analysis was carried out using the SPSS software (version 22.0). Enumeration data were expressed as numbers or percentages (%) and measured by chi-square test or Fisher's exact test. Measurement data were expressed as (*x̅*±sd) and measured by independent samples *t*-test. Kaplan-Meier method was used to analysis RFS of patients in each group. Fisher's exact test was utilized to compare 1-year, 2-year, and 3-year IS recurrence rates between the two groups. The level of statistical significance was set at *p* < 0.05.

## 3. Results

### 3.1. Baseline Information

Baseline information of patients in two groups was collected and analyzed for comparison. The results displayed no significant difference in sex, age, body mass index (BMI), past medical history (hypertension, diabetes, hyperlipidemia), smoking history, alcoholism history, and drug regimen (*p* > 0.05). In addition, comparisons in cholesterol level (TC, TG, LDL-C, HDL-C) of patients in two groups revealed that the difference (*p* = 0.081, *p* = 0.175, *p* = 0.939, *p* = 0.403) was not statistically significant at baseline level (see Table 1).

### 3.2. Evaluation Indicators of Success of LAAO in Treating Patients in the Observation Group

Patients in the observation group were reexamined by TEE 45 d and 6 months after LAAO to measure whether there was residual shunt in the LAA and thrombosis on surface of the occluder. Forty-five d after LAAO, TEE suggested that 50% of patients (30/60) had complete occlusion of LAA, with 51.7% (31/60) patients having residual shunt ≤ 5 mm. Six months after LAAO, TEE suggested that 58.3% of patients (35/60) had complete occlusion of LAA, with 15.0% (9/60) of patients having residual shunt ≤ 5 mm. Taken together, all occluders met the efficacious occluding criteria during follow-up visits of 45 d and 6 months (see Table 2).

### 3.3. Comparison of Recurrence of IS and Incidence of Systemic Embolism of Patients between Two Groups

Incidence of systemic embolism in the observation group (1.67%, 1/60) was markedly lower than that in the control group (13.33%, 11/60), with the difference presenting statistical significance (*p* = 0.014). IS recurrence in the observation group (3.33%, 2/60) was significantly lower than that in the control group (18.33%, 11/60), with the difference presenting statistical significance (*p* = 0.008). Details are listed in Table 3.

### 3.4. Comparison of RFS of Patients between Two Groups

The average RFS in the control group was 29.91 months (95% CI: 27.50~32.31 months) and that in the observation group was 31.97 months (95% CI: 29.85~32.92 months). The differences in two groups presented statistical significance (*p* < 0.05) (Figure 1). Comparison of 3-year IS recurrence between two groups was shown in Table 4. The differences of 1-year recurrence rate (*p* = 0.014), 2-year recurrence rate (*p* = 0.008), and 3-year recurrence rate (*p* =0.008) all reached statistical significant. These results demonstrated that LAAO could effectively prolong RFS of patients with previous IS.

## 4. Discussion

IS, responsible for permanent disability in adults in most cases, is the second common cause of dementia, with mortality of patients ranking third globally [18]. Compelling evidence exists that 5-year recurrence rate of IS is up to 18% [19]. Oral anticoagulants (warfarin or novel oral anticoagulants) have been widely applied to IS treatment, but their clinical application is limited since long-term usage increases the risk of bleeding in patients [20]. LAAO can efficaciously prevent thrombi in LAA from joining into blood circulation and reduce risk of IS. As such, this study indicated that patients with previous IS undergoing LAAO had lower disease recurrence rate and longer RFS when compared to those without LAAO.

Patients in the observation group were reexamined by TEE 45 d and 6 months later to measure whether there was residual shunt in the LAA and thrombosis on surface of the occluder. The results of TEE showed that complete occlusion of LAA was found in 50% of patients (30/60) in the observation group 45 d later while it was found in 58.3% of patients (35/60) 6 months later, suggesting that all occluders met the efficacious occluding criteria. These results are similar to findings of Boersma et al. [21] that success rate of LAAO arises from 90.9% in PROTECT AF to 95.1% in PREVAIL and 98.5% in EWOLUTION, suggestive of high implant and block success rate of LAAO. In this study, the Watchman occluder was used for patients in the observation group. It is a self-expanding nitinol occlusion device surrounded with barbs, and the other side is covered with a polytetrafluoroethylene (PTFE) porous membrane ensuring free blood flow in and out of LAA [22, 23].

Roman-Gonzalez et al. [24] proposed that patients with IS are resistant to aspirin, which is implicated with IS recurrence. Earlier investigations believed that LAAO is an efficacious preventive therapy for thrombosis, especially for patients with previous IS, and a warfarin contraindication or advanced age [13]. Phillips et al. [25] carried out a study on 201 patients with nonvalvular atrial fibrillation undergoing LAAO, and after the procedure, they are prescribed novel oral anticoagulant. After 2 years of follow-up, incidence rates of IS and bleeding are 1.9% and 2.2%, respectively, 77% and 49% reductions versus those as expected, indicating that LAAO has a long-term effect in preventing IS in patients with atrial fibrillation. Another study also illustrated that LAAO has a high success rate and a low incidence of complications in clinical application [26]. LAAO is a novel alternative for patients with high risk of IS recurrence who are poorly responded to anticoagulants. As such, this study revealed that recurrence of IS and incidence of systemic embolism of patients in the observation group were lower than those in the control group, suggesting that LAAO may reduce the recurrence rate of IS and the occurrence of systemic thrombotic events, which is similar to results by Fink et al. [27]. Comparison of 3-year RFS between two groups revealed that RFS of patients in the observation group was notably longer than that in the control group. The median survival time of the observation group was 31.97 months, and the median survival time of the control group was 29.91 months. Collectively, LAAO for patients with prior IS could effectively decrease recurrence of IS and prolong RFS of patients, thus improving their survival quality. In addition, LAAO also brings some risks of complications. For instance, a study [28] pointed out that LAAO may cause occluder-related thrombosis. Nevertheless, this is a retrospective study; therefore, incidence of occluder-related thrombotic complications is not fully recorded. The small sample size is another limitation. It is necessary to expand the sample size and to provide clinical trials with higher evidence levels for verification of safety and effectiveness of LAAO in preventing IS recurrence.

In summary, regarding patients with prior IS who had poor therapeutic responses to thrombolytics and anticoagulants, LAAO could effectively decrease recurrence of IS and incidence of systemic embolism, thus prolonging RFS of patients. LAAO also found to be highly efficacious. It was, therefore, an alternative method for patients with high risk of IS recurrence.

## Figures and Tables

**Figure 1:** RFS of patients in two groups.

**Table 1:** Baseline information.

Baseline information	Control group (*n* = 60)	Observation group (*n* = 60)	*χ*2/*t*	*p* value
Age (year)	55.90 ± 10.44	57.19 ± 9.63	0.702	0.484
Sex			0.141	0.707
Male	36	38		
Female	24	22		
BMI (kg/m^2^)	24.70 ± 1.78	25.34 ± 2.23	1.722	0.088
Past medical history (yes)				
Hypertension	18	24	1.319	0.251
Diabetes	14	12	0.196	0.658
Hyperlipidemia	9	11	0.240	0.624
Smoking history			0.315	0.575
Yes	35	38		
No	25	22		
Alcoholism history			0.302	0.583
Yes	29	26		
No	31	34		
Drug regimen				
Antiplatelet drugs	21	24	0.320	0.572
Statins	23	19	0.586	0.444
Anticoagulants	18	21	0.342	0.559
Cholesterol level				
TC	6.13 ± 0.55	6.33 ± 0.65	1.762	0.081
TG	2.39 ± 0.65	2.56 ± 0.72	1.366	0.175
LDL-C	4.14 ± 0.93	4.12 ± 1.03	0.076	0.939
HDL-C	1.61 ± 0.36	1.68 ± 0.55	0.839	0.403

TC: total cholesterol; TG: triglyceride; LDL-C: low-density lipoprotein cholesterol; HDL-C: high-density lipoprotein cholesterol.

**Table 2:** Evaluation indicators of success of LAAO in treating patients in the observation group.

TEE test time	Complete occlusion of LAA	Residual shunt ≤ 5 mm
45 d	50.0% (30/60)	51.7% (31/60)
6 months	58.3% (35/60)	15.0% (9/60)

TEE: transesophageal echocardiography.

**Table 3:** Comparison of recurrence of IS and incidence of systemic embolism of patients between two groups.

Indicator	Control group (*n* = 60)	Observation group (*n* = 60)	*χ*2	*p* value
Incidence of systemic embolism	13.33% (8/60)	1.67% (1/60)	6.018	0.014
Recurrence of IS	18.33% (11/60)	3.33% (2/60)	6.988	0.008

**Table 4:** Comparison of 3-year IS recurrence of patients between two groups.

IS recurrence	Control group (*n* = 60)	Observation group (*n* = 60)	*χ*2	*p* value
1-year recurrence	10.00% (6/60)	0.00% (0/60)	6.316	0.014
2-year recurrence	18.33% (11/60)	3.33% (2/60)	6.988	0.008
3-year recurrence	18.33% (11/60)	3.33% (2/60)	6.988	0.008

## Data Availability

The data that support the findings of this study are available on request from the corresponding author.
